This article has been retracted.

# Prediction Model of Ischemic Stroke Recurrence Using PSO-LSTM in Mobile Medical Monitoring System

**DOI:** 10.1155/2022/8936103

**Published:** 2022-03-24

**Authors:** Qingjiang Li, Xuejiao Chai, Chunqing Zhang, Xinjia Wang, Wenhui Ma

**Affiliations:** ^1^School of Medical Technology, Qiqihar Medical University, Qiqihar, Heilongjiang 161000, China; ^2^School of Public Health, Qiqihar Medical University, Qiqihar, Heilongjiang 161000, China; ^3^Clinical Teaching Center, Qiqihar Medical University, Qiqihar, Heilongjiang 161000, China; ^4^School of General Practice and Continuing, Qiqihar Medical University, Qiqihar, Heilongjiang 161000, China

## Abstract

Aiming at the problems of low prediction accuracy and low sensitivity of traditional ischemic stroke recurrence prediction methods, which limits its application range, by introducing an adaptive particle swarm optimization (PSO) algorithm into the Long and Short-Term Memory (LSTM) model, a prediction model of ischemic stroke recurrence using deep learning in mobile medical monitoring system is proposed. First, based on the clustering idea, the particles are divided into local optimal particles and ordinary particles according to the characteristic information and distribution of different particles. By updating the particles with different strategies, the diversity of the population is improved and the problem of local optimal solution is eliminated. Then, by introducing the adaptive PSO algorithm into the LSTM, the PSO-LSTM prediction model is constructed. The optimal super parameters of the model are determined quickly and accurately, and the model is trained combined with the patient's clinical data. Finally, by using SMOTE method to process the original data, the imbalance of positive and negative sample data is eliminated. Under the same conditions, the proposed PSO-LSTM prediction model is compared with two traditional LSTM models. The results show that the prediction accuracy of PSO-LSTM model is 92.0%, which is better than two comparison models. The effective prediction of ischemic stroke recurrence is realized.

## 1. Introduction

Researches show that the death caused by cerebrovascular diseases ranks first and second among the causes of death in China. The incidence rate of ischemic stroke accounts for more than 75% of cerebrovascular diseases [1]. In recent years, advanced technologies such as deep learning methods and mobile medical monitoring have been developed and widely applied in medicine. In response to the high incidence rate, high mortality rate, and high recurrence rate of ischemic stroke, the coping strategies gradually changed from treatment-based to prediction-based [2, 3]. Early recurrence prediction and effective response measures for cerebrovascular diseases are the key factors for the prevention and treatment of stroke recurrence, which is also the focus of research in the medical industry [4–6].

At present, more than 94% of ischemic stroke is caused by specific and controllable factors such as lifestyle, hypertension, and aging [7, 8]. Therefore, the incidence rate and mortality rate of ischemic stroke patients can be significantly decreased according to the main causes and current physiological state of ischemic stroke [9, 10]. In [11], elderly patients, who had early transient ischemic attack and had a poor prognosis, were divided into recurrence group and nonrecurrence group. The criterion for judging the poor prognosis was whether there was recurrence one month after the onset. According to logistic regression analysis, the clinical characteristics of the two groups were compared, and a guiding method that can predict the recurrence of ischemic stroke was proposed. However, this method only analyzes the characteristics after the early onset of the disease, which has some limitations. Reference [12] took patients with depression and cerebrovascular diseases as the research object and used the diagnosis of depression as the index date to track and record the recurrence of cerebrovascular diseases. The results showed that the risk of cerebrovascular diseases recurrence mainly depends on age and physical health but had little relationship with depression and psychotropic drugs. This method mainly analyzed the effect of depression on the recurrence of cerebrovascular diseases but did not give the specific factors affecting the recurrence of cerebrovascular diseases. The results of [13] showed that asymptomatic cerebral infarction is an independent predictive factor of clinical cerebrovascular events and can be used as a prediction index of cerebrovascular events recurrence to predict ischemic stroke. However, this method only proves the predictive effect of asymptomatic cerebral infarction on cerebrovascular diseases and cannot be applied to most patients. Reference [14] obtained relevant feature information by learning the clinical characteristics of stroke patients using the bidirectional LSTM method and enhanced the utilization efficiency of index information according to the attention mechanism. The authors proposed a risk prediction model of ischemic stroke based on the bidirectional LSTM (BiLSTM) network and attention mechanism. However, this method does not classify the clinical characteristics of patients in detail, and the prediction accuracy is not optimal. Reference [15] obtained the patient's characteristic information by learning the electronic medical record of patients with cardiovascular and cerebrovascular diseases using the Recurrent Neural Network (RNN), proposed a cardiovascular and cerebrovascular disease risk prediction model based on electronic medical record data mining, and improved the prediction accuracy of the model by fusing various types of clinical data. However, this method does not consider the difference of pathogenesis in different patients, and there are some defects. Reference [16] designed the embolization mechanism of Shuxuetong injection in prevention of acute ischemic stroke recurrence and carried out relevant experiments. The experimental results provided an effective basis for the effectiveness and safety of Shuxuetong injection in reducing stroke recurrence in patients with ischemic stroke. However, this method only studied and verified the preventive effect of Shuxuetong injection and did not put forward a substantive prediction basis. Reference [17] scored patients with acute ischemic stroke based on Cox regression analysis, divided the risk of ischemic stroke recurrence under different scores by establishing a scoring mechanism, and realized the prediction of ischemic stroke recurrence by calibrating and distinguishing the scores. However, the score of this method has not been fully verified when applied to external data sets and has poor prediction accuracy.

Based on the above analysis, aiming at the problems of small application scope and low accuracy of most existing ischemic stroke recurrence prediction methods, an ischemic stroke recurrence prediction model using deep learning in mobile medical monitoring system is proposed. The adaptive PSO algorithm can improve the population diversity and solve the problem of falling into the local optimal solution. It can effectively predict the recurrence of ischemic stroke by introducing PSO into LSTM and combining the patient's clinical data.

## 2. Model Establishment

### 2.1. Problem Description

The recurrence prediction of ischemic stroke can be mathematically described as the feature mapping relationship between the prediction index of the current time or a future time *t* and the corresponding label.

For the historical data of *h* patients, set the prediction index data set as *A*={*a*_1_, *a*_2_, *a*_3_,…, *a*_*h*_} and the label set corresponding to the data set as *B*={*b*_1_, *b*_2_, *b*_3_,…, *b*_*h*_}. On the basis of constructing the prediction model of ischemic stroke recurrence, the feature mapping relationship between the prediction index data set *A* and the corresponding label set *B* is obtained by training the model. According to the obtained feature mapping relationship between the prediction data and the corresponding label, for the newly emerging patients outside the label set, based on the patient's prediction data, the optimal risk prediction result *B*′={*b*_1_′, *b*_2_′, *b*_3_′,…, *b*_*h*_′} is obtained through the ischemic stroke recurrence prediction model.

### 2.2. LSTM Neural Network Prediction Model of Adaptive PSO

#### 2.2.1. PSO Algorithm of Adaptive Learning Strategy

The establishment of the prediction model is based on the adaptive PSO algorithm, and the traditional adaptive PSO algorithm is improved by introducing LSTM to construct the ischemic stroke recurrence prediction model. It can use the PSO algorithm of adaptive learning strategy to match the data features of ischemic stroke patients with the topology of LSTM neural network, so as to achieve higher prediction performance.

In order to improve the diversity of the initial population as much as possible, the clustering idea is the basic idea in the process of model construction. First, based on the feature information of different particles in the particle swarm and their respective distribution, the whole particle swarm is divided into multiple subgroups with different features. Then, different learning strategies are adopted for different subgroups to improve the diversity of the whole population [18].

The process of dividing particle swarm is based on simplified PSO algorithm and simplified PSO algorithm with extreme value disturbance [19]. The algorithms can automatically obtain the cluster center of the sample data set and can realize high-performance clustering and fast search for any shape of data. The basic basis is that the cluster center contains two basic features surrounded by points with low local density, and the information of the two features is far away from the points with high local density. The basic principle is as follows:

If there is a population *E* in the search space of *W* dimension, and the population is composed of *e* particles, the population *E* can be expressed as *E*={*l*_*k*_}_*k*=1_^*e*^, where *l*_*k*_ represents the *k*-th particle in the population *E*, which contains *W* dimensions and can be expressed as *l*_*k*_={*l*_*k*1_, *l*_*k*2_, *l*_*k*3_,…, *l*_*kW*_}. Two variables are given from the *w*-th dimension of the *k*-th particle: local density and distance. The local density of the particle is defined as *ρ*_*kw*_, and its expression is as formula (1):

(1) $$\begin{array}{c} \rho_{kw}=\sum_{k\neq j}\exp\left[-\frac{D_{kj}{}^{2}}{D_{T}}\right], \end{array}$$

where *D*_*kj*_ represents the Euclidean distance between the *k*-th particle and the *j*-th particle. *D*_*T*_ represents the truncation distance.

The distance between the *k*-th particle and the *j*-th particle with higher local density is defined as *σ*_*kw*_, and its expression is as follows:

(2) $$\begin{array}{c} \sigma_{kw}=\underset{j:\rho_{jw}>\rho_{kw}}{\min}\left\{D_{kj}\right\}. \end{array}$$

For the sample data with the largest local density *ρ*_*kw*_, the value of *σ*_*kw*_ is $\underset{j}{\max}\left\{D_{kj}\right\}$.

As can be seen from formula (2), if the density of *l*_*kw*_ is the maximum local density, *σ*_*kw*_ will be much greater than the distance *σ* of its nearest particle. Therefore, the center of each divided subgroup is generally some particles with very large *σ*, and the local density *ρ* of these particles is also relatively large. When selecting the cluster centers for different subgroups, particles with relatively large distance *σ* and local density *ρ* can be selected. For the particles other than the cluster center, according to the *l*_*jw*_ of the particle, the particle can be divided into subgroups where the sample with local density greater than *l*_*jw*_ and closest to *l*_*jw*_ is located.

After the overall division of particle swarm, according to the division results of subgroups, the particles in each subgroup are reclassified into two categories: locally optimal particles and ordinary particles, and they are iteratively updated by different update methods to achieve the purpose of increasing population diversity.

Ordinary particles expand the local search ability under the guidance of the optimal particle and update iteratively based on

(3) $$\begin{array}{c} l_{kw}=\alpha \cdot l_{kw}+\beta_{1}R_{1w}\left(L_{\text{PO}kw}-l_{kw}\right)+\beta_{2}R_{2w}\left(I_{\text{PO}kw}-l_{kw}\right). \end{array}$$

In formula (3), *α* represents the inertia weight coefficient. *β*_1_ and *β*_2_ represent learning factors. *R*_1*w*_ and *R*_2*w*_ represent random numbers which obey uniform distribution in the interval [0,1]. *L*_PO*kw*_ represents the optimal position information of the *w*-th dimension of the *k*-th particle. *I*_PO*kw*_ represents the optimal location information in the *i*-th subgroup.

For locally optimal particles, in order to strengthen the information interaction between different subgroups, they are generally updated by collecting the information of different subgroups. The update process is shown in formula (4).

(4) $$\begin{array}{c} l_{kw}=\alpha \cdot l_{kw}+\beta_{1}R_{1w}\left(L_{\text{PO}kw}-l_{kw}\right)+\beta_{2}R_{2w}\left(\frac{1}{I}\sum_{i=1}^{I}I_{\text{PO}kw}-l_{kw}\right). \end{array}$$

In formula (4), *I* represents the total number of subgroups.

From the above analysis, it can be seen that, in a certain subgroup, the main function of local optimal particles is to guide the search direction of the whole subgroup. They can not only guide other ordinary particles to learn, but also undertake the task of information exchange between different subgroups. If the local optimal particle updates with the same update strategy as other ordinary particles, the local optimal particle will lose the ability to interact with other subgroups, and its search direction is likely to deviate from the optimal search direction. At this time, the subgroup will fall into the trap of local optimal solution. Therefore, the local optimal particle needs to break through the constraints of the subgroup and interact with other subgroups in the process of updating, so as to ensure the correctness of the search direction by obtaining effective information from other subgroups, as shown in (4). In this way, information sharing among different subgroups can improve population diversity.

#### 2.2.2. PSO-LSTM Prediction Model

The clinical data of patients with ischemic stroke can be regarded as a time series. There are many factors inducing their disease recurrence, and all the factors are very complex, uncertain, nonlinear, and unstable [20]. In order to accurately predict the factors inducing disease recurrence to the greatest extent, a prediction model for ischemic stroke recurrence is constructed based on LSTM according to the common features of time series.

The network structure of LSTM is mainly affected by some parameters in the model [21]. In order to make LSTM more suitable for the prediction of ischemic stroke recurrence, a new LSTM ischemic stroke recurrence prediction model based on PSO algorithm is constructed by fusing and optimizing the adaptive PSO algorithm and LSTM.

It can be seen from the previous analysis that the adaptive PSO algorithm has many unique advantages, such as simple algorithm design, fast calculation speed, and convergence speed, and makes up for the defect that it is easy for the ordinary PSO algorithm to fall into the trap of local optimal solution. The adaptive PSO algorithm greatly improves the performance in finding the optimal solution [22]. PSO algorithm combined with LSTM can quickly and accurately determine the optimal super parameters and finally realize the effective prediction of ischemic stroke recurrence.

The basic structure of LSTM ischemic stroke recurrence prediction model based on PSO algorithm is shown in Figure 1 below.

The model construction process mainly includes the following steps:

(1) The adaptive PSO algorithm is used to optimize some parameters of LSTM, including time window parameters, the number of hidden layer units, and batch processing parameters. The position information of different particles in particle swarm optimization is initialized based on the value range of super parameters.
(2) Based on local density of the particle *ρ*_*kw*_ and the distance *σ*_*kw*_ between this particle and the particle with higher local density calculated by formulas (1) and (2), finally, the adaptive partition of particle swarm is realized, and several subgroups are obtained.
(3) Based on the super parameter value corresponding to the particle position information, the LSTM is constructed. The training data are used to learn and train the constructed model. Then use the validation data to predict and verify the trained LSTM.
(4) Construct fitness values for particles. The definition of fitness function is shown in formula (5), which is the average absolute percentage error of the model on the validation data set.
  (5) $$\begin{array}{c} F=\frac{1}{S_{v}}\sum_{i=1}^{S_{v}}\frac{\left|n_{i}^{\prime }-n_{i}\right|}{n_{i}}. \end{array}$$
In formula (5), *S*_*v*_ represents the total amount of data in the validation data set. *n*_*i*_′ represents the predicted value of the *i*-th validation data. *n*_*i*_ represents the true value of the *i*-th validation data.
(5) The fitness values of particles in all different subgroups are calculated, and based on their fitness values, these particles are divided into ordinary particles, subgroup optimal particles, and global optimal particles. On this basis, for different classes of particles, their position information is calculated and updated with the formulas shown in equations (3) and (4).
(6) Determine whether to terminate the calculation. If the termination conditions are met, it means that the global optimal solution of the optimization objective has been obtained. If the termination conditions are not met, the subpopulation should be regrouped according to the updated particle position information, and steps 2–5 should be repeated until the termination conditions are met. The global optimal solution of the super parameter is obtained.
(7) The LSTM is constructed according to the global optimal solution of the obtained hyperparameters, and the model is trained and predicted based on the clinical data of patients with ischemic stroke.

## 3. Prediction of Ischemic Stroke Recurrence

### 3.1. Multifactor Determination

Because the factors affecting the recurrence of ischemic stroke are very complex, it is necessary to screen the relevant indicators. In the medical field, logistic regression analysis is usually widely used to analyze and study the causal relationship between independent variables and dependent variables [23]. Next, logistic regression analysis is used to analyze and determine the multiple factors affecting the recurrence of ischemic stroke. The dependence between independent variables and dependent variables can be characterized by regression coefficients, and the calculation of regression coefficients can be obtained by calculating category probability [24]. The calculation methods of category probability and regression coefficient are shown in formulas (6) and (7), respectively.

(6) $$\begin{array}{c} P\left(b=c|a\right)=\frac{\exp\left[\eta_{c}+\sum_{m=1}^{M}\lambda_{cm}a_{m}\right]}{1+\sum_{c=1}^{C-1}\left(\eta_{c}+\lambda_{cM}a_{M}\right)}, \end{array}$$

(7) $$\begin{array}{c} \ln\left[\frac{P\left(b=c|a\right)}{P\left(b=C|a\right)}\right]=\eta_{c}+\sum_{m=1}^{M}\lambda_{cm}a_{m}. \end{array}$$

In formulas (6) and (7), *a* represents the independent variable. *c* represents the dependent variable. *M* represents the number of independent variables.

When *M*=1, there is only one independent variable. At this time, the model carries out single factor analysis to analyze the impact of a single independent variable on the dependent variable. When *M* > 1, the number of independent variables is more than one; the model carries out multifactor analysis to analyze the comprehensive impact on the dependent variables when multiple independent variables change at the same time. Finally, the model comprehensively analyzes the risk factors of ischemic stroke recurrence by changing the number of independent variables.

### 3.2. Determination of Input and Output Variables

According to the problem description, the main problem to be solved in constructing the prediction model of ischemic stroke recurrence is the feature mapping relationship between the prediction index data set *A* and the corresponding label set *B*, that is, the feature mapping relationship between input variables and output variables. In order to predict the recurrence of ischemic stroke, firstly, it should be clear whether the input variables and output variables meet the requirements of the model. Given two data sets *D*={(*d*_*i*(*t* − 1)_, *d*_*it*_)}_*i*=1_^*h*^ and *G*={*g*_*i*_ ∈ {0,1}}, where *i* represents the *i*-th patient, *d*_*i*(*t* − 1)_ represents the predictive index data of the *i*-th patient at the time *t* − 1 and contains a group of multiple incentives affecting the recurrence of ischemic stroke. *G* represents the diagnostic label of each sample.

The following is an analysis of the input variable (the prediction data set *A*) and the output variable (the corresponding label set *B*).

(1) The input variable (the prediction data set *A*)
First, the LSTM ischemic stroke recurrence prediction model based on PSO algorithm is calculated through the determined *d*. For the *i*-th patient, based on the data index *d*_*t*−1_ of the current time *t* − 1, the change *d*_*t*_′ of the continuous value in the data index *d*_*t*_ of the future time *t* is fitted. The fitting process is shown as follows.
  (8) $$\begin{array}{c} d_{it}^{\prime }=\mu \left[\text{PSO}-\text{LSTM}\left(d_{i\left(t-1\right)},d_{it}\right)\right]. \end{array}$$
On this basis, the data indexes of time *t* − 1 and time *t* are combined to form the prediction index data input variable *A*, as follows.
  (9) $$\begin{array}{c} A=\text{concat}\left[d_{i\left(t-1\right)},d_{it}^{\prime }\right]. \end{array}$$
(2) The output variable (the corresponding label set *B*)

For the *i*-th patient, the real label set *B* of the patient is obtained by converting the obtained sample diagnostic label *G* into a one-dimensional array, as follows.

(10) $$\begin{array}{c} B=\left\{b_{1},b_{2},b_{3},\ldots ,b_{h}\right\}. \end{array}$$

In formula (10), *b*_*i*_ ∈ *g*_*i*_, *i*=1,2,…, *h*.

After obtaining the prediction index data set *A* and the corresponding label set *B*, the proposed prediction model searches the feature mapping relationship between *A* and *B* and finally obtains the prediction results of ischemic stroke recurrence risk, as shown in formula (11).

(11) $$\begin{array}{c} B^{\prime }=\text{soft}\max\left[\text{LSTM}\left(A,B\right)\right]. \end{array}$$

### 3.3. Data Acquisition and Preprocessing

Before using LSTM ischemic stroke recurrence prediction model based on PSO algorithm to predict the recurrence risk, it is necessary to collect patient data and preprocess these data.

Data collection is mainly carried out through the big data management platform for stroke patients. The platform is mainly based on data access and import tools. It takes the medical institutions, sanitary places, healthcare institutions, physical examination centers, and institutions of various hospitals scattered all over the country as the collection objects and collects the source data of different stroke patients. Finally, a uniquely researchable and structured patient case information database about stroke patients was formed [25]. Data collection for patients mainly includes the following aspects: Personal information, past medical history, family history, laboratory data, inpatient diagnosis and treatment data, periodic follow-up data and physical examination data, etc. The data import tool of the platform can provide a compatible heterogeneous data acquisition interface for different types of stroke heterogeneous data sources and can import data from a variety of relational databases from different patients and institutions. In terms of data acquisition strategy, the data import tool of the platform can realize the access and import of full, batch, and real-time data. For offline data, the platform can also import log data files such as HDFS, FTP, and text files. In addition, it can also import streaming data such as Flume and Kafka in real time.

The purpose of data preprocessing is to clean, interpolate missing values, eliminate abnormal data, and standardize data format and other operations for the source data of stroke patients with complex, extensive, and diverse data forms and types. Data preprocessing unifies the data format of stroke patients to improve the overall data quality to a certain extent [26]. On this basis, the influencing factors of ischemic stroke are assigned as the independent variables of modeling. Finally, these data are more suitable for the requirements of model construction.

### 3.4. Model Training

In order to find the best model parameter, in the process of training the model, the calculation error is calculated by calculating the loss function at each step, and on this basis, the optimizer is used for reverse adjustment and update.

In the binary classification loss problem, the cross-entropy loss function is widely used to calculate the loss. It can reflect the effect of model training by calculating the error between the predicted value and the real label. The cross-entropy loss function is shown in formula (12).

(12) $$\begin{array}{c} F_{\text{Lce}}=-\sum_{i=1}^{h}b_{i}\log\left(b_{i}^{\prime }\right). \end{array}$$

In formula (12), *h* represents the total number of sample data.

The difference between the probability of ischemic stroke recurrence *b*_*i*_′ and the real label *b*_*i*_ was calculated by maximum likelihood operation.

In the process of reverse adjustment and update using the optimizer, in order to reduce the loss of model training and avoid falling into the trap of local optimal solution, Adam optimizer is used for reverse calculation to adjust the weight parameters of the network. On this basis, the adaptive learning rate is designed by calculating the first-order moment estimation and second-order moment estimation of the gradient.

The gradient ∇*t* at time *t* is calculated based on the loss function *F*_*Lt*_ of the target. The calculation process is shown in formula (13).

(13) $$\begin{array}{c} \nabla t⟵\Delta_{\gamma }F_{Lt}\left(\gamma_{t-1}\right). \end{array}$$

In formula (13), *γ* represents the update parameter corrected by moment estimation.

According to the gradient ∇*t* at time *t* calculated by formula (13), the first-order and second-order moment estimates *m*_1*t*_ and *m*_2*t*_ are calculated. The calculation process is shown in formulas (14) and (15), respectively.

(14) $$\begin{array}{c} m_{1t}⟵\xi_{1}m_{1t-1}+\left(1-\xi_{1}\right)\nabla t, \end{array}$$

(15) $$\begin{array}{c} m_{2t}⟵\xi_{2}m_{2t-1}+\left(1-\xi_{2}\right)\nabla t^{2}. \end{array}$$

In formulas (14) and (15), *ξ*_1_ and *ξ*_2_ represent the attenuation index of moment estimation, and their values are *ξ*_1_=0.900 and *ξ*_2_=0.999.

## 4. Experiments and Analysis

### 4.1. Parameter Setting

The parameters of the model are set before the experiment. The proposed PSO-LSTM model in this paper mainly includes four parts: the input layer, the first LSTM layer, the second LSTM layer, and the output layer. The loss function adopts the cross-entropy loss function, the optimizer adopts the Adam algorithm optimizer, and the construction of the network model is completed based on the Keras framework. The super parameters in LSTM model mainly include time window size, batch size, training times, and the number of neurons in hidden layer.

In order to minimize the error and influence of human factors on the model as much as possible, four super parameters in the LSTM model are set based on the clinical data of actual ischemic stroke patients, which are as follows: the value range of time window size is set to [1,20], the value range of batch size is set to [1,60], and the value range of the number of neurons in the hidden layer is set to [10,30]. The training times are mainly determined by the loss of the model. Since the loss function of the model will gradually converge after 500 iterations, the training time of the model is 500. In addition, other relevant parameters are set as follows: the total number of particles in the particle swarm is set to 50, the maximum number of iterations is set to 300, the inertia weight of velocity is set to *α*=0.85, and the sum of acceleration coefficient is set to 1.8.

### 4.2. Evaluation Index

In order to effectively measure the accuracy of LSTM ischemic stroke recurrence prediction model based on PSO algorithm, the following five evaluation indexes are used to evaluate the experimental results.

(1) Accuracy: the calculation method is
  (16) $$\begin{array}{c} E_{a}=\frac{S_{TT}+S_{FF}}{S_{TT}+S_{TF}+S_{FT}+S_{FF}}. \end{array}$$
(2) Sensitivity: the calculation method is
  (17) $$\begin{array}{c} E_{se}=\frac{S_{TT}}{S_{FT}+S_{FF}}. \end{array}$$
(3) Specificity: the calculation method is
  (18) $$\begin{array}{c} E_{sp}=\frac{S_{FF}}{S_{FT}+S_{FF}}. \end{array}$$
(4) Positive prediction rate: it is calculated as follows:
  (19) $$\begin{array}{c} E_{p}=\frac{S_{TT}}{S_{TT}+S_{FT}}. \end{array}$$
(5) Negative prediction rate: it is calculated as follows:
  (20) $$\begin{array}{c} E_{n}=\frac{S_{FF}}{S_{TF}+S_{FF}}. \end{array}$$
(6) F1_score: the calculation method is shown in the following equation:

(21) $$\begin{array}{c} E_{F1}=\frac{2E_{p}\cdot E_{se}}{E_{p}+E_{se}}. \end{array}$$

In formulas (15)–(21), *S*_*TT*_ represents the number of patients who are actually with recurrent ischemic stroke and are correctly predicted as the patients with recurrent ischemic stroke. *S*_*TF*_ indicates the number of patients who are actually with recurrent ischemic stroke but are incorrectly predicted as patients without recurrent ischemic stroke. *S*_*FT*_ indicates the number of patients who are not with recurrent ischemic stroke but are incorrectly predicted as patients with recurrent ischemic stroke. *S*_*FF*_ indicates the number of patients who are not with recurrent ischemic stroke and are correctly predicted as patients without recurrent ischemic stroke.

### 4.3. Normalization

During the experiment, the clinical data of all ischemic stroke patients, i.e., the input sample values, were normalized to compress the values within the value range [0,1] [27]. Next, it takes 2000 total cholesterol concentration sample data as an example for normalization. The numerical changes of sample data before and after normalization are shown in Figure 2.

It can be seen from Figure 2 that, after normalization, the total cholesterol concentration of the sample data is compressed from [0,18] to [0,1] on the basis of maintaining the basic characteristics of the original data.

### 4.4. Experimental Results

In order to eliminate the influence caused by the imbalance of positive and negative sample data in the process of data collection, the collected sample data are balanced by Synthetic Minority Oversampling Technique (SMOTE). The data processed by SMOTE method not only solves the problem of data imbalance between positive and negative samples but also expands the diversity of data samples to a certain extent. The calculation results of different evaluation indexes before and after SMOTE method are shown in Table 1 below.

It can be seen from Table 1 that, compared with the results of ischemic stroke recurrence prediction using the original data, the accuracy, sensitivity, specificity, positive prediction rate, negative prediction rate, and F1_score of recurrence prediction using the data processed by SMOTE method have improved. The prediction accuracy reached 92%, with a relative increase of 14%. In addition, it can be seen that, before using SMOTE method to process the data, the specificity of the prediction results is 81%, the sensitivity is 69%, and the difference between them is 12%, which shows that the negative sample has more feature information than the positive sample in the data used in the learning process of the model, and there are more omissions in predicting the recurrence of ischemic stroke patients. The positive prediction rate is 62% and the negative prediction rate is 86%, with a difference of 24%, which shows that the model has a high probability of misjudgment in the prediction process. When the SMOTE method is used to process the data, the specificity of the prediction results is 90%, and the sensitivity is 91%. They are basically the same. The positive prediction rate is 85%, and the negative prediction rate is 83%. They are also basically the same. The test results of positive and negative samples have been significantly improved and achieved a relatively balanced effect.

Next, the prediction results of PSO-LSTM ischemic stroke recurrence prediction model proposed in this paper are compared with the prediction methods proposed in [14, 15]. The prediction results are shown in Table 2 below.

It can be seen from Table 2 that the accuracy of PSO-LSTM ischemic stroke recurrence prediction model proposed in this paper is 92.0%, which is improved compared with the other two prediction models. The sensitivity and specificity of the other two prediction models are lower than that of PSO-LSTM model. This is because the model proposed in [14] has relatively poor learning ability for time-series feature data set. Reference [15] does not introduce attention mechanism, while PSO-LSTM model assigns corresponding attention weight to each time-series feature, so the sensitivity and specificity of the model have been improved. In addition, it can be seen that the positive prediction rate and negative prediction rate of the prediction results of PSO-LSTM model are relatively high. This is because the adaptive PSO optimization algorithm is not introduced in [14, 15], and the introduction of PSO can reduce the prediction omission in the prediction process. In addition, SMOTE method is used to process the sample data, which eliminates the imbalance of positive and negative sample data and makes F1_score increase.

In order to better illustrate the consistency between the prediction results of PSO-LSTM ischemic stroke recurrence prediction model proposed in this paper and the actual results, the receiver operating characteristic (ROC) curve of the model is analyzed below. The ROC curve of PSO-LSTM prediction model is shown in Figure 3.

As can be seen from Figure 3, the ROC curve of PSO-LSTM prediction model is relatively far from the 45° classifier baseline with discrimination of 0, and the lower area of ROC curve reaches 0.89, which shows that PSO-LSTM prediction model has strong discrimination and good performance. By introducing the adaptive PSO algorithm into LSTM, the rapid determination of the optimal super parameters is realized based on the historical characteristics of patient clinical data. By using SMOTE method to process the original data, the effective prediction of ischemic stroke recurrence is realized and the prediction accuracy is improved.

## 5. Conclusion

According to the historical clinical data of ischemic stroke patients, reasonable prediction of stroke recurrence can effectively reduce the mortality of patients. Therefore, an ischemic stroke recurrence prediction model using deep learning in mobile medical monitoring system is proposed by introducing adaptive PSO algorithm into LSTM. In order to solve the clustering and searching problem of the existing prediction models for the clinical data of stroke patients, the proposed model introduces adaptive learning strategy based on PSO algorithm. By dividing the types and update methods of particles, it avoids the possibility of falling into local optimization on the basis of improving the diversity of the population and improves the clustering performance and searching speed of the model. Experiments based on the data from big data management platform for stroke patients show that the accuracy of PSO-LSTM ischemic stroke recurrence prediction model proposed in this paper is 92% and F1_score is 88%, which are better than the prediction performance of the other two models. In addition, the sensitivity and specificity, positive prediction rate, and negative prediction rate of PSO-LSTM prediction model are improved compared with the other two models, and the lower area of ROC curve reaches 0.89, which has better performance. Future work will further study the prediction effect of the proposed PSO-LSTM prediction model on patients with ischemic stroke and other types of diseases and study the performances of different diseases on the prediction model.

## Figures and Tables

**Figure 1:** The structure of the LSTM ischemic stroke recurrence prediction model based on adaptive PSO.

**Figure 2:** Sample data before and after normalization. (a) Initial source data. (b) Normalized data.

**Figure 3:** ROC curve of PSO-LSTM prediction model.

**Table 1:** Calculation results of different evaluation indexes before and after processing by SMOTE method.

Evaluation index	Before SMOTE processing (%)	After SMOTE processing (%)
Accuracy (*E*_a_)	78.2	92.0
Sensitivity (*E*_se_)	69.3	91.2
Specificity (*E*_sp_)	81.1	90.5
Positive prediction rate (*E*_p_)	62.6	85.3
Negative prediction rate (*E*_n_)	86.4	83.7
F1_score (*E*_F1_)	65.8	88.5

**Table 2:** Evaluation indexes for prediction results of different methods.

Evaluation index	Model		
	PSO-LSTM (%)	Reference [14]	Reference [15]
Accuracy (*E*_a_)	92.0	86.2	85.1
Sensitivity (*E*_se_)	91.2	84.4	83.5
Specificity (*E*_sp_)	90.5	82.2	80.1
Positive prediction rate (*E*_p_)	85.3	82.6	83.1
Negative prediction rate (*E*_n_)	83.7	80.7	80.2
F1_score (*E*_F1_)	88.5	82.5	81.9

## Data Availability

The data included in this paper are available without any restriction.
